This article has been retracted.

# Mini-plate versus Kirschner wire internal fixation for treatment of metacarpal and phalangeal fractures in Chinese Han population: a meta-analysis

**DOI:** 10.1186/1749-799X-9-24

**Published:** 2014-04-11

**Authors:** Jiaming Xu, Changqing Zhang

**Affiliations:** 1 Department of Orthopedics, Shanghai Jiaotong University Affiliated Sixth People's Hospital, 600 Yishan Road, Shanghai, Shanghai Province 200233, China

**Keywords:** Mini-plate internal fixation, Kirschner wire, Chinese Han population, Metacarpal/phalangeal fracture, Meta-analysis

## Abstract

**Objectives:**

This meta-analysis aimed to compare the therapeutic effect of mini-plate versus Kirschner wire (K-wire) internal fixation on the treatment of metacarpal and phalangeal fractures among Chinese Han population.

**Methods:**

Databases of China National Knowledge Infrastructure (CNKI), Wanfang, Chinese VIP, PubMed, and Embase were retrieved for studies on mini-plate (case group) versus K-wire (control group) internal fixation for the treatment of metacarpal and phalangeal fractures among Chinese Han population. The odds ratio (OR) and standardized mean difference (SMD) at 95% confidence interval (CI) were used for estimating the effects of dichotomous data and continuous data, respectively. All statistical analyses were performed by Review Manager 5.2 software.

**Results:**

A total of 18 studies involving 1,375 metacarpal or phalangeal fracture patients (709 cases and 666 controls) were included in the meta-analysis. There were significant differences in fracture healing time (SMD = −1.28; 95% CI: −1.81, −0.76), postoperative infection rate (OR = 0.25; 95% CI: 0.16, 0.39), complication incidence (OR = 0.24; 95% CI: 0.15, 0.38), and surgery time (SMD = 1.57; 95% CI: 0.76, 2.37) between the case and the control group, while no significant difference was found in hospital stays between these two groups (SMD = 0.43; 95% CI: −0.34, 1.20; *P* = 0.27).

**Conclusions:**

For the treatment of metacarpal or phalangeal fracture among Chinese Han population, mini-plate has advantages of shorter healing time and lower infection rate and complication incidence compared with K-wire internal fixation, while a longer surgery time than K-wire. In conclusion, mini-plate is prior than K-wire internal fixation for the treatment of metacarpal or phalangeal fracture among Chinese Han population.

## Introduction

Metacarpal/phalangeal are injury-prone in daily work and life. Metacarpal and phalangeal fractures constitute 10% of all fractures [1]. Due to the complex structure and special function of the hand, the treatment has always been one of the intricate problems in orthopedic physicians. The metacarpal/phalangeal fractures are often treated with closed reduction with internal fixation (CRIF).

CRIF has been widely used to treat the majority of unstable closed simple hand fractures [2] and has been a mainstay of treatment for most phalangeal fractures [3] since the percutaneous screws and Kirschner wire (K-wire) were introduced a method of CRIF [4]. However, because of the less rigid fixation with little stability of the K-wire, it is limited in the treatment of unstable fractures, while mini-plate is considered as a potential option for unstable fractures of the hand with good stability allowing early mobilization of joints and avoiding problems associated with protruding K-wire [5-7].

At present, in China, both mini-plate internal fixation and K-wire internal fixation are commonly used. Plenty of clinical studies compared the outcomes (operative time, hospital stay, fracture healing time, and incidence of postoperative complications) of these two methods for the treatment of metacarpal/phalangeal fracture [8-25]. However, most of the studies were with low sample numbers, and the results were inconsistent. Therefore, in this study, we performed a meta-analysis by comprehensively evaluating the published medical evidences to compare the effect of mini-plate internal fixation and K-wire.

## Materials and methods

### Search strategy

The China National Knowledge Infrastructure (CNKI) database (http://www.cnki.net/), Chinese Wanfang database (http://www.wanfangdata.com.cn/), Chinese VIP database (http://www.cqvip.com/), PubMed (http://www.ncbi.nlm.nih.gov/pubmed), and Embase (http://www.elsevier.com/online-tools/embase) were retrieved independently by two investigators for eligible studies published before November 2013. The keywords included metacarpal/phalangeal fracture, mini-plate internal fixation, Kirschner wire, and Han/Chinese/China.

### The eligible criteria

Inclusion criteria were as follows: (1) the study was designed as randomized controlled trials or retrospective case-control study; (2) the study compared the effect of mini-plate fixation with K-wire fixation for the treatment of metacarpal and phalangeal fractures; (3) patients were adults (≥18 years old); (4) the outcomes contained at least one evaluation: fracture healing time, operative time, hospital stay, postoperative infection, and incidence of postoperative complications; and (5) the study provided enough information for pooled evaluation of each effect indicator.

Exclusion criteria were as follows: (1) the study with incomplete data or duplication was excluded, and (2) review articles, letters, and comments were also excluded.

### Data extraction and quality assessment

Two investigators independently evaluated each included studies for extraction of the relevant characteristics including the first author, publication year, region of study origin, sample size, number of patients with mini-plate or K-wire internal fixation, general demographic data (e.g., the proportion of gender, age in the experimental group and control group), the outcome measures (fracture healing time, operation time, length of hospital stay, postoperative infection, the incidence of postoperative complications). If there were any disputes in the process of data extraction, a third evaluator joined for group discussions and referencing to the original study. The quality evaluation of included studies was assessed by Jadad scale [26]. Studies with 0–2 points were divided into low-quality documents, and those with 3–5 points were considered high-quality documents.

### Statistical analysis

Meta-analysis was performed by Review Manager 5.2 software. The heterogeneity among included studies was evaluated by *Q* statistics [27] and *I*^*2*^ test. *P* > 0.05 and/or *I*^*2*^ < 50% was considered no significant heterogeneity, and a fixed effects model was used for calculating the pooled effect size. Otherwise, the random effects model was used. For the continuous data, the standardized mean difference (SMD) and 95% confidence interval (CI) were used to estimate the effects of each outcome, while for dichotomous data and continuous data, the odds ratio (OR) and 95% CI were used. The publication bias was estimated by Begg's funnel plot test. A thorough sensitivity analysis was performed to assess the robustness of combined estimates to different assumptions and inclusion criteria [28].

## Results

### The characteristics of the included studies

A total of 936 documents were obtained by computer retrieval of the databases according to the search strategy. The literature screening process was listed in Figure 1. By screening the title and abstracts, 891 documents were excluded, and then by reviewing of the full text, 18 articles with insufficient data and 9 duplications were excluded. Finally, a total of 18 studies [8-25] including 1,375 cases were included in this meta-analysis. There were 709 patients in the case group (mini-plate) and 666 patients in the control group (K-wire). The characteristics of the included studies were listed in Table 1. By Jadad scale quality assessment, the included studies were all low-quality documents with 1–2 points because most of the included studies did not report the random allocation methods.

**Figure 1:** The flow diagram of literature screening process.

**Table 1:** The characteristics of the included studies

**Author**	**Year**	**Region**	**Case/control**			**Outcomes**	**Score**
			***n***	**Male (%)**	**Age**		
Chu FZ	2008	Jilin	43/51	73.2	31.4	a	1
Duan YZ	2006	Henan	25/31	76/65.7	23.4/22.3	de	1
Huang CY	2007	Guangxi	40/40	82.5/87.5	31.6/29.1	d	1
Jin DF	2012	Hubei	46/44	73.9/72.7	37.5/39.5	abcde	1
Li HF	2012	Hebei	39/39	71.8/74.4	33.5/33.2	abd	2
Li JT	2013	Ningxia	51/38	66.7/68.4	37.6/36.1	abcd	1
Lin CX	2008	Zhejiang	33/22	60.6/68.2	33.4/35.4	d	1
Lu LM	2013	Jiangsu	34/34	55.9/58.8	35.2/36.2	abc	2
Ma HZ	2012	Ningxia	58/55	77.9	31	ade	2
Qiuj Z	2009	Sichuan	42/35	64.3/62.9	33.5/34.6	abcd	2
Tang SY	2004	Guangdong	50/41	73.6	23.4	ade	2
Wang JL	2011	Neimenggu	43/43	-	-	ade	2
Wang MZ	2011	Heilongjiang	38/38	60.5	35	de	1
Wu H	2012	Hubei	45/33	70.1	32.6	abcde	2
Xu HD	2012	Jiangsu	20/20	-	-	ae	1
Yang JG	2013	Guangdong	36/36	61.1/63.9	34.8/35.1	abcd	2
Yang JJ	2011	Guangdong	34/34	61.8/64.7	34.2/34.1	abcd	2
Zhou B	2010	Guangdong	32/32	75	37.3	abcde	2

*a* the fracture healing time, *b* the surgery time, *c* duration of hospital stay, *d* infection rate, *e* incidences of complication. Score, the points of Jadad quality assessment of the included studies.

### Heterogeneity test

No significant heterogeneity was found among studies of the infection rate (Figure 2), so the fixed effects model was used for pooling of the effect size. While there were significant heterogeneities in fracture healing time, operation time, length of hospital stay (Table 2), and the incidence of postoperative complications (Figure 3) among the studies, thus the random effects models were used for pooled analysis of these indicators.

**Figure 2:** The forest plot of infection rate.

**Table 2:** **The meta**-**analysis results of fracture healing time**, **surgery time**, **and duration of hospital stay**

**Outcomes**	**Northern China**		**Southern China**		**Total**		**Heterogeneity**	
	***n***	**SMD (95% CI)**	***n***	**SMD (95% CI)**	***n***	**SMD (95% CI)**	***P***	***I***^**2 **^**(%)**
Fracture healing time	7	−2.05 (−3.01, −1.08)	7	−0.57 (−0.95, −0.19)	14	−1.28 (−1.81, −0.76)	<0.00001	94
Surgery time	3	5.83 (2.33, 9.34)	6	0.74 (0.43, 1.05)	9	1.57 (0.76, 2.37)	<0.00001	96
Duration of hospital stay	2	2.15 (−2.26, 6.56)	6	−0.09 (−0.52, 0.35)	8	0.43 (−0.34, 1.20)	<0.00001	95

**Figure 3:** The forest plot of postoperative complication rate.

### Outcome measures

To minimize the influence of region, subgroup analysis was conducted by dividing the data to northern China and southern China.

#### Infection rate

The infection rate in the case group was significantly lower than that in the control group. The OR of infection rate was 0.27 (95% CI: 0.13, 0.59) among northern Chinese population and 0.24 (95% CI: 0.14, 0.42) among southern Chinese population. The pooled OR was 0.25 (95% CI: 0.16, 0.39) in Chinese population (Figure 2).

#### Fracture healing time

The healing time in the case group was significantly shorter than that in the control group. The SMD of fracture healing time was −2.05 (95% CI: −3.01, −1.08) and −0.57 (95% CI: −0.95, −0.19) in northern China and southern China, respectively, and the pooled SMD was −1.28 (95% CI: −1.81, −0.76) (Table 2).

#### Surgery time

The surgery time in the case group was significantly longer than that in the control group. The SMD of fracture healing time was 5.83 (95% CI: 2.33, 9.34) and 0.74 (95% CI: 0.43, 1.05) in northern China and southern China, respectively, and the pooled SMD was 1.57 (95% CI: 0.76, 2.37) (Table 2).

#### Duration of hospital stay

There was no significant difference in duration of hospital stay between the case and the control group. The SMD of duration of hospital stay was 2.15 (95% CI: −2.26, 6.56) and −0.09 (95% CI: −0.52, 0.35) in northern China and southern China, respectively, and the pooled SMD was 0.43 (95% CI: −0.34, 1.20) (Table 2).

#### Postoperative complications

The incidence of postoperative complication in the case group was significantly shorter than that in the control group. The OR of postoperative complications was 0.25 (95% CI: 0.12, 0.50) and 0.71 (95% CI: 0.10, 5.28) in northern China and southern China, respectively, and the pooled OR was 0.38 (95% CI: 0.14, 1.05) (Figure 3).

#### Publication bias estimate

Begg's funnel plot test was performed to estimate the publication bias. The funnel plots of postoperative infection rates and incidence of postoperative complications between the case group and the control group are shown in Figures 4 and 5, respectively. The shapes of the two funnel plots were symmetrical, indicating no significant publication bias among the included studies.

**Figure 4:** The funnel plot of infection rate.

**Figure 5:** The funnel plot of complication incidence.

#### Sensitivity analysis

Sensitivity analysis was performed for measuring the effects of the omitted study which may largely influence the overall pooled OR [29]. By sensitivity analysis, the results of fracture healing time, operative time, hospital stay, and postoperative infection rates were all robust. While for incidence of postoperative complications, Jin's study [11] was found to be highly influential. After excluding this study, the OR of postoperative complication incidence was 0.22 (95% CI: 0.11, 0.45) and 0.25 (95% CI: 0.13, 0.48) in northern China and southern China, respectively, and the pooled OR was 0.24 (95% CI: 0.15, 0.38) (Figure 6). These results indicate that the mini-plate is superior to K-wire internal fixation for the treatment of metacarpal and phalangeal fractures.

**Figure 6:** The forest plot of postoperative complication rate after sensitivity analysis.

## Discussion

To our knowledge, this study is the first meta-analysis to explore the effect of mini-plate fixation compared with K-wire fixation of metacarpal and phalangeal fractures in Chinese Han population and draws significant conclusions. The results of this meta-analysis, involving 1,375 patients (mini-plate for 709 patients, K-wire for 666 patients), are consistent with the conclusions of most previous clinical or retrospective studies [8-25] that the mini-plate fixation is superior to K-wire fixation in the treatment of metacarpal and phalangeal fractures.

K-wire fixation is simple to manipulate and without or with little damage on fracture blood supply, and has been used extensively. Since in the K-wire fixation there is no compression on the fracture [30], it is difficult to control the motions of the fingers. In some cases, it is necessary to pass the K-wire through the metacarpophalangeal or interphalangeal joint and externally fixed with plaster after the operation [31]. This is not conducive to the early motions of the hand joints and is prone to cause complications such as infection, stiffness, and malunion, as well as delay of fracture healing [32]. Mini-plate fixation is more stable and allows the straightaway motion of the finger [31,33], which is conducive to reduce the complications and expedite the fracture healing. In the present study, mini-plate showed advantages of lower infection rate (OR = 0.25; 95% CI: 0.16, 0.39), lower complication incidence (OR = 0.38; 95% CI: 0.14, 1.05), and shorter healing time (SMD = −1.28; 95% CI: −1.81, −0.76) compared with the K-wire. However, the mini-plate also showed disadvantage of relatively difficult procedure and high costs and invasiveness [33]. In addition, longer surgery time was found in patients treated with mini-plate fixation than K-wire (SMD = 1.57; 95% CI: 0.76, 2.37; *P* < 0.05) in the present study.

To avoid influences of confounding factors, we restricted our study to the Chinese Han population, and all subjects of the included documents are Chinese Han ancestry. There was no statistical heterogeneity among the results of postoperative infection rates and incidence of postoperative complications. However, China is a vast country; therefore, the regional and cultural differences and clinical levels may result in the heterogeneity in meta-analysis of fracture healing time, operation time, and length of stay of indicators. Although we conducted stratified analysis by dividing Chinese Han population into southern China and northern China by region to make findings more reliable, heterogeneity still existed in these three indicators. Due to the incomplete information about the relevant covariates such as patient gender and age of patients, types of devices, and the postoperative medical care in the selected literature, some other potential confounding factors were not taken into account in the present meta-analysis. Additionally, the quality of the included studies in the present meta-analysis was not high, which may also influence the results of the present study. Therefore, more well-designed clinical studies with high quality are essential in the future.

## Conclusions

The present meta-analysis indicated that the mini-plate fixation was more suitable than the K-wire fixation for the treatment of metacarpal and phalangeal fractures among the Chinese Han population when considering the healing time, postoperative infection, complications, and hospital stays. However, more large-scale independent studies are essential to validate the findings of this study in the future.

## Abbreviations

CRIF: closed reduction with internal fixation; K-wire: Kirschner wire; CNKI: China National Knowledge Infrastructure; SMD: standardized mean difference; CI: confidence interval; OR: odds ratio.

## Competing interests

The authors declare that they have no competing interests.

## Authors' contributions

JX and CZ drafted the manuscript. CZ carried out the immunoassays. JX participated in the sequence alignment. JX participated in the design of the study and performed the statistical analysis. CZ conceived of the study and participated in its design and coordination and helped draft the manuscript. Both authors read and approved the final manuscript.
